This article has been retracted.

# Construction and Evaluation of Neural Network Correlation Model between Syndrome Elements and Physical and Chemical Indexes of Unstable Angina Pectoris Complicated with Anxiety

**DOI:** 10.1155/2022/6217186

**Published:** 2022-08-21

**Authors:** Xiaoyang Chen, Yifei Wang, Li Zhang, Xuegong Xu

**Affiliations:** ^1^Guangzhou University of Chinese Medicine, Guangzhou 510016, China; ^2^Henan University of Chinese Medicine, Zhengzhou 450046, China; ^3^Cardiovascular department, Zhengzhou Hospital of Chinese Medicine, Zhengzhou 450007, China; ^4^Laboratory of Zhengzhou Hospital of Traditional Chinese Medicine, Zhengzhou 450007, China; ^5^Key Laboratory of traditional Chinese medicine for cardiovascular diseases of Henan Province, Zhengzhou 450007, China

## Abstract

**Objective:**

Syndrome elements are regarded as the smallest unit of syndrome differentiation, which is characterized by indivisibility and random combination. Therefore, it can well fit the goal of syndrome differentiation and unity.

**Methods:**

Clinical physicochemical indicators are important references for disease diagnosis, but they are often not used too much in the process of TCM syndrome differentiation. In the era of intelligence, communicating TCM syndrome differentiation at the macro level with physiological and pathological processes at the micro level (i.e., these clinical physicochemical indicators) is an effective tool to realize intelligent medicine. Taking the collected relevant clinical physical and chemical indexes as the research object, on the basis of routine *t*-test and nonparametric test, logistic regression model is used to mine the main syndrome elements, and neural network multilayer perceptron is used to predict the feature model.

**Results:**

Compared with non-blood stasis patients, there were significant differences in HGB, PLT, Pt, PTA, Na^+^, TG, LDL, BNP, LVEDd, and EF in blood stasis patients. Taking blood stasis as the dependent variable and the above physical and chemical indexes with statistical significance (*P* < 0.05) as independent variables. Compared with non-qi depression patients, there were significant differences in atpp, TG, TC, LDL, LVESD, and FS in qi depression patients (*P* < 0.05). Taking Yin deficiency as dependent variable and the above physical and chemical indexes (Hgb, APTT, CKMB, LVEDd, and LVPW) with statistical significance (*P* < 0.05) as independent variables, binary logistic regression analysis was carried out.

**Conclusion:**

The combination pattern of physical and chemical indexes obtained from the neural network model provides a clinical reference basis for identifying the syndrome elements of unstable angina pectoris complicated with anxiety, such as blood stasis, qi depression, Qi deficiency, yin deficiency, phlegm turbidity, and qi stagnation.

## 1. Background

Chinese medicine has remarkable curative effect in the treatment of patients with heart disease. Traditional Chinese medicine (TCM) has apparent advantages in stabilizing the heart disease, improving heart function, and improving the quality of life. In recent years, inspired by modern medicine, many doctors try to explain the mechanism of syndrome with a single experimental index in order to solve the problem of syndrome inconsistency. Because syndrome is the overall response of multiple system levels [1], the results often have certain limitations. Although it can show its relevance, it is difficult to justify it in the process of interpretation.

Syndrome elements are regarded as the smallest unit of syndrome differentiation, which is characterized by indivisibility and random combination [2]. It is the key to realize the objectification of syndrome [3], so it can well fit the goal of syndrome differentiation and unity. Clinical physicochemical indicators are important references for disease diagnosis, but they are often not used too much in the process of TCM syndrome differentiation [4]. In today's intelligent era, communicating TCM syndrome differentiation at the macro level with physiological and pathological processes at the micro level (i.e., these clinical physicochemical indicators) is an effective tool to realize intelligent medicine [5]. In the face of the regularity of TCM syndromes and the multilevel problems of pathophysiology, data mining technology shows great advantages. Through literature search, no research on the combination of macro and micro was found.

Therefore, based on the syndrome related data collected in the process of clinical epidemiological investigation, this study explored the distribution and combination characteristics of TCM syndrome elements in unstable angina pectoris complicated with anxiety and provides reference for the unity of syndrome differentiation of the disease. Then, taking the collected relevant clinical physical and chemical indexes as the research object, on the basis of routine *t*-test and nonparametric test, logistic regression model is used to mine the main syndrome elements, neural network multilayer perceptron is used to predict the characteristic model, and the correlation between the main syndrome elements and physical and chemical indexes of unstable angina pectoris complicated with anxiety is analyzed to explore the role and significance of the combination mode of clinical physical and chemical indexes in the diagnosis of syndrome elements.

## 2. Materials and Methods

### 2.1. Observation Object

The cases came from patients hospitalized in the Department of Cardiology of Zhengzhou hospital of traditional Chinese medicine from January 2017 to January 2019. Our study was approved by the institutional review board of the hospital, and written informed consent was obtained from each participant.

### 2.2. Diagnostic Criteria of Western Medicine

Diagnostic criteria of unstable angina pectoris: refer to the 2016 guidelines for the diagnosis and treatment of unstable angina pectoris and non-ST segment elevation myocardial infarction. Diagnostic criteria of anxiety state: Under the guidance of psychiatrists, all patients were scored and investigated with HAMA anxiety scale. Specific criteria: ≥29 points are classified as severe anxiety state; ≥21 points, obvious anxiety; ≥14 points, there must be anxiety; ≥7 points, may have anxiety; and <7 points, no anxiety.

### 2.3. Diagnostic Criteria of TCM Syndrome Elements

Referring to the relevant parts in terms of clinical diagnosis and treatment of traditional Chinese medicine syndrome [6] in 1997 and the guiding principles for clinical research of new traditional Chinese medicine, diagnostics of traditional Chinese medicine, and internal medicine of traditional Chinese medicine in 2002, it is divided into blood stasis, phlegm turbidity, cold coagulation, yin deficiency, Qi deficiency, Yang deficiency, qi stagnation, excess dampness, fire heat, and qi depression. Within 24 hours of admission, three deputy directors or above, clinicians with relevant clinical experience of 5 years or above and trained will judge the syndrome elements on the basis of disease diagnosis. The criteria for determining the patient's syndrome elements are as follows: ① when the opinions of 3 clinicians are consistent; ② if the opinions of two clinicians are consistent with that of another clinician, the first two opinions shall be adopted; ③ if the opinions of the three clinicians are inconsistent, the doctors with the qualification of deputy director and above shall re-collect the information of the four diagnoses and re-judge the syndrome elements until they meet the conditions of ① and ②.

### 2.4. Inclusion Criteria

The inclusion criteria are as follows: (1) 18-79 years old; (2) unstable angina pectoris; (3) HAMA anxiety was between 14 and 29 points; (4) normal cognitive function and no reading and writing impairment; and (5) after informed consent, they can voluntarily cooperate and participate in the investigation and research.

### 2.5. Exclusion criteria

The exclusion criteria are as follows: (1) severe valvular disease, cardiomyopathy, pericardial disease, congenital heart disease, cardiogenic shock, acute myocarditis, infective endocarditis, and severe arrhythmia with hemodynamic changes; (2) other congenital diseases such as rheumatic aortic stenosis and syphilis; (3) liver dysfunction (liver function index value >2 times the normal value) and renal insufficiency (renal insufficiency decompensated period, CCR <50 ml/min, SCR >2 mg/dL, or >177 *μ*Mol/L), serious electrolyte disorders, blood system and other primary diseases, malignant tumors, pulmonary embolism, diabetes combined with severe complications, hypertension, hyperthyroidism, hypothyroidism, and other serious endocrine diseases or other uncontrollable systemic diseases; and (4) pregnant or lactating women.

### 2.6. Removal, Falling Off, and Suspension Standards

These are enumerated as follows: (1) patients who were wrongly included, (2) patients whose data were incomplete for various reasons after inclusion and could not be counted; and (3) patients who were unable to complete the study due to mental or physical disorders.

### 2.7. Collection of Clinical Routine Indexes

All selected patients completed white blood cell (WBC), red blood cell (RBC), hemoglobin concentration (HGB), platelet (PLT), thyroglobulin (TG), total cholesterol (TC), high density lipoprotein cholesterol (HDL), low density lipoprotein cholesterol (LDL), cardiac troponin (cTnI), myoglobin, CKMB, alt, AST, bun within 1-3 days after admission creatinine (CR), N-terminal pro-B-type natriuretic peptide (NT proBNP), potassium (K+), sodium (Na+), chloride (Cl-), calcium (Ca2+), prothrombin time (PT), prothrombin activity (PTA), partial prothrombin time (APTT), fibrinogen concentration (FIB), D-dimer (D-D), left ventricular end diastolic diameter (LVEDd), left ventricular end systolic diameter (LVESD), left ventricular posterior wall thickness (LVPW), ventricular septal thickness (IVS), left ventricular stroke output (SV), output per minute (CO), left ventricular end diastolic volume (EDV), left ventricular end systolic volume (ESV), ejection fraction (EF), left ventricular short axis shortening rate (FS), left atrial inner diameter (LAD), right ventricular inner diameter (RIV), and other examinations. Fill in the results in the clinical information collection form and attach relevant copies.

### 2.8. Neural Network Model Construction Method

The dependent variable is a binary variable. Binary logistic regression square analysis is used to assign values to the dependent variable, in which “yes =1” and “no =0.” The method is forward: Wald (forward stepwise method). The test level of the variable entering the model is less than 0.05. Taking the physical and chemical indexes (*P* < 0.05) entered into logistic in each syndrome element as the covariate and each syndrome element as the dependent variable; a neural network model was established and tested.

### 2.9. Statistical Methods

SPSS21.0 for statistical analysis of data was used. The measurement data of normal distribution is described by (± s), and the counting index is described by frequency and composition ratio. For the hypothesis test of comparison between the two groups, the measurement data of normal distribution adopts *t*-test, the counting data adopts C2 test, and the measurement data of non-normal distribution adopts rank sum test. According to international standards, there was significant difference (*P* < 0.05).

## 3. Result

### 3.1. General Information

From January 2017 to January 2019, 238 eligible cases were collected in the inpatient department of Cardiology of Zhengzhou hospital of traditional Chinese medicine, of which 13 cases were excluded because the score of HAMA anxiety scale was between 7 and 14; 6 cases were excluded due to lack of blood lipid index test results; 11 cases were excluded due to lack of cardiac color Doppler ultrasound results; and 8 cases were excluded due to lack of liver and kidney function test results. There were 137 more women, with a constituent ratio of 68.5%. The average age of the patients was 59.77 ± 10.79, the minimum age was 33 years old, and the maximum age was 79 years old. Most of the patients were between 51 and 70 years old, accounting for 59.0%. The majority of patients were retired, followed by workers and intellectuals. The most common syndrome elements are blood stasis, accounting for 84.5%, followed by qi depression, a total of 137 cases, accounting for 68.5%, followed by qi deficiency and yin deficiency, accounting for 47.0% and 42.5%, respectively, followed by phlegm turbidity and qi stagnation, accounting for 27.0% and 26.0%, with less heat accumulation, Yang deficiency, dampness, and cold coagulation.

### 3.2. Factor Screening of Physical and Chemical Indexes Related to Syndrome Elements

#### 3.2.1. Blood Stasis

Due to the small number of cases of heat accumulation, excessive dampness, Yang deficiency, and cold coagulation, it will not be discussed in the correlation analysis. By nonparametric test or *t*-test, compared with nonblood stasis patients, there were significant differences in HGB, PLT, Pt, PTA, Na^+^, TG, LDL, BNP, LVEDd, and EF in blood stasis patients (*P* < 0.05), as shown in Table 1.

Taking blood stasis as the dependent variable and the above physical and chemical indexes (Hgb, PLT, Pt, PTA, Na^+^, TG, LDL, BNP, LVEDd, and EF) with statistical significance (*P* < 0.05) as independent variables, binary logistic regression analysis is carried out. The results are shown in Table 2. Four indexes enter the regression equation, namely, HGB, Pt, PTA, and ef (*P* < 0.05), as shown in Table 2.

#### 3.2.2. Qi Depression

Compared with non-qi depression patients, there were significant differences in atpp, TG, TC, LDL, LVESD, and FS in qi depression patients (*P* < 0.05), as shown in Table 3.

Taking qi depression as the dependent variable and the above physical and chemical indexes (atpp, TG, TC, LDL, LVESD, and FS) with statistical significance (*P* < 0.05) as independent variables, binary logistic regression analysis was carried out. As shown in Table 4, the three indexes entered the regression equation, namely, APTT, TC, and FS (*P* < 0.05), as shown in Table 4.

#### 3.2.3. Qi Deficiency

Compared with non-Qi deficiency patients, the differences of HGB, APTT, K +, BNP, LVEDd, and LAD in Qi deficiency patients were statistically significant (*P* < 0.05), as shown in Table 5.

Taking Qi deficiency as the dependent variable and the above physical and chemical indexes with statistical significance (*P* < 0.05) (Hgb, APTT, K +, BNP, LVEDd, and LAD) as independent variables, binary logistic regression analysis was carried out. As shown in Table 6, the three indexes entered the regression equation, namely, HGB, LVEDd, and LAD (*P* < 0.05), as shown in Table 6.

#### 3.2.4. Yin Deficiency

Compared with non-Yin deficiency, HGB, APTT, CKMB, LVEDd, and LVPW in patients with Yin deficiency were statistically significant (*P* < 0.05), as shown in Table 7.

Taking Yin deficiency as dependent variable and the above physical and chemical indexes (Hgb, APTT, CKMB, LVEDd, and LVPW) with statistical significance (*P* < 0.05) as independent variables, binary logistic regression analysis was carried out. As shown in Table 8, four indexes entered the regression equation, namely, APTT, CKMB, LVEDd, and LVPW (*P* < 0.05), as shown in Table 8.

#### 3.2.5. Phlegm Turbidity

Compared with non-phlegm turbidity, the differences of HGB, PLT, APTT, alt, AST, Cl-, LVEDd, and FS in patients with phlegm turbidity were statistically significant (*P* < 0.05), as shown in Table 9.

Taking phlegm turbidity as dependent variable and the above physical and chemical indexes (Hgb, PLT, APTT, alt, AST, Cl-, LVEDd, and FS) with statistical significance (*P* < 0.05) as independent variables, binary logistic regression analysis was carried out. As shown in Table 10, four indexes entered the regression equation, alt, APTT, LVEDd, and FS (*P* < 0.05), as shown in Table 10.

#### 3.2.6. Qi Stagnation

Compared with non-qi stagnation, the differences of WBC, HGB, Pt, FIB, HDL, BNP, LVEDd, and LAD in Qi stagnation patients were statistically significant (*P* < 0.05), as shown in Table 11.

The above physical and chemical indexes (WBC, HGB, Pt, FIB, HDL, BNP, LVEDd, and LAD) with statistical significance (*P* < 0.05) were taken as independent variables for binary logistic regression analysis. As shown in Table 12, six indexes entered the regression equation, namely, WBC, Pt, BNP, FIB, LVEDd, and lad, as shown in Table 12.

### 3.3. Construction and Evaluation of Neural Network Model

Taking blood stasis as dependent variable and HGB, Pt, PTA, and EF as covariates, build a neural network model and test the model. The results are shown in Figure 1. The accuracy of the model is 85.4% in the training set and 87.1% in the test set.

Taking qi depression as the dependent variable and APTT, TC, and FS as the covariates, the neural network model is established and tested. The results are shown in Figure 2. The accuracy of the model is 71.1% in the training set and 69.0% in the test set.

Taking Qi deficiency as the dependent variable and HGB, LVEDd, and lad as covariates, the neural network model is established and tested. The results are shown in Figure 3. The accuracy of the model is 88.8% in the training set and 91.2% in the test set.

Taking Yin deficiency as dependent variable and APTT, CKMB, LVEDd, and LVPW as covariates, a neural network model is built and tested. The results are shown in Figure 4. The accuracy of the model is 75.0% in the training set and 75.0% in the test set.

Taking phlegm turbidity as dependent variable and alt, APTT, LVEDdm and FS as covariates, build a neural network model and test the model. The results are shown in Figure 5. The accuracy of the model is 79.8% in the training set and 73.2% in the test set.

Taking qi stagnation as the dependent variable and WBC, Pt, BNP, FIB, LVEDd, and lad as the covariates, the neural network mode is established, and the model is tested. The results are shown in Figure 6. The accuracy of the model is 82.6% in the training set and 79.0% in the test set.

## 4. Discussion

Unstable angina pectoris complicated with anxiety has the common characteristics of unstable angina pectoris and anxiety. Literature studies have found that the most common syndrome elements of coronary heart disease complicated with anxiety are qi stagnation, blood stasis, phlegm, and heat accumulation. In this study, blood stasis, qi depression, Qi deficiency, yin deficiency, phlegm turbidity, and qi stagnation are the most common syndrome elements, which is generally consistent with the results of literature research.

From the perspective of syndrome combination, the syndrome types of three factor combination and four factor combination appear more in this study, and the syndrome performance tends to be complex. In the combination of syndromes, other syndromes are mainly superimposed on the basis of qi depression and blood stasis, suggesting that qi depression and blood stasis are the key pathogenesis of the disease and the main pathological link. However, blood stasis syndrome accounts for 84.5% of the total cases, indicating that blood stasis is the initiating factor of the occurrence of the disease. As the “syndrome sanctions” says: “the depression within the seven emotions starts with Qi injury, and the blood will follow.”

HGB is a protein, whose main function is to transport oxygen. It combines with oxygen in the lungs, then transports it to various tissues and organs of the whole body, and transports the waste away at the same time [7]. After anemia, the myocardium is in a state of hypoxia. If the body itself suffers from coronary heart disease, it will increase the burden of the heart, resulting in myocardial ischemia and hypoxia. The patient will show an increase in the number of angina pectoris attacks [8], the aggravation of the degree of angina pectoris, and then develop into heart failure and blood stasis [9]. In this study, HGB in patients was lower than that in non-deficiency and blood stasis group. It is considered that patients in blood stasis group may have anemia.

FS is an index parameter of left ventricular systolic function. It is a sensitive index reflecting myocardial contractility. Its calculation is the ratio of the shortening value of left ventricular diameter at each contraction to the ventricular diameter at each end of diastole. Studies have shown that there is an obvious linear correlation between FS and EF and FS is more accurate and repeatable than EF in evaluating cardiac systolic function [10]. In this study, the level of FS is high, suggesting that compared with patients with non-qi depression syndrome, the myocardial contractility of patients with qi depression syndrome may be relatively better.

Studies have shown that lad can accurately predict the mortality of patients with coronary heart disease and heart failure [11]. The enlargement of LAD reflects a certain degree of myocardial remodeling. When the left ventricular systolic function is not changed, the increase of LAD reflects the impairment of left ventricular diastolic function [12]. Studies have shown that the increase of lad is comparable to the decrease of LVEF [13]. In this study, lad in patients with Qi deficiency syndrome is relatively high, suggesting that patients with Qi deficiency syndrome may have certain myocardial remodeling and reduced systolic function.

ALT is an important raw material for the synthesis of a variety of non-essential amino acids. It is involved in the diagnosis of many diseases. The liver is the most common site of alt, followed by the kidney, heart, and skeletal muscle. ALT includes the following: two isozymes, alts, and ALTM, exist in cytoplasm and mitochondria, respectively, and the activity of the latter is greater than that of the former. The increase of serum ALT generally indicates liver injury, and the damaged hepatocytes are mainly ALTM [14], while the serum ALT is low, and the disease is generally not considered. In this study, the ALT level of phlegm turbidity syndrome is lower than that of non-phlegm turbidity syndrome, and there are few studies on this aspect. Therefore, the relationship between phlegm turbidity syndrome and ALT still needs to be discussed.

FIB is a “protagonist” protein synthesized by the liver and playing a role in the coagulation system. It is a class II glycosylated protein synthesized by the liver and free in plasma. Its half-life is 3-6 days, and its molecular metabolic rate is 31-46 mg/kg. It accounts for about 3% of the total plasma protein [15]. When coagulation occurs, FIB is hydrolyzed into fibrin monomer under the action of thrombin and then cross-linked to fibrin. In addition, FIB can specifically bind to platelet membrane glycoprotein II B/III a receptor to promote platelet aggregation^1, 2^ [16, 17]. In this study, FIB in patients with qi stagnation syndrome was significantly lower than that in patients with non-qi stagnation syndrome, suggesting that the blood coagulation function of patients with qi stagnation syndrome was reduced. However, this study also has some shortcomings, such as not including the number of cases in a wider range and not using external validation set validation. Besides, the mechanism is not verified. Further studies are needed to study this.

## 5. Conclusion

To sum up, the combination pattern of physical and chemical indexes obtained from the neural network model provides a clinical reference basis for identifying the syndrome elements of unstable angina pectoris complicated with anxiety, such as blood stasis, qi depression, Qi deficiency, yin deficiency, phlegm turbidity, and qi stagnation.

## Figures and Tables

**Figure 1:** Neural network model for distinguishing blood stasis by characteristic indexes.

**Figure 2:** Neural network model for distinguishing qi depression by characteristic indexes.

**Figure 3:** Neural network model for distinguishing Qi deficiency by characteristic indexes.

**Figure 4:** Neural network model for distinguishing Yin deficiency by characteristic indexes.

**Figure 5:** Neural network model for distinguishing phlegm turbidity by characteristic indexes.

**Figure 6:** Neural network model for distinguishing qi stagnation by characteristic indexes.

**Table 1:** Factors of physical and chemical indexes related to blood stasis.

	Blood stasis (*n* = 169)	Non-blood stasis (*n* = 31)	*P*
HGB(g/L)	120.07 ± 22.18	128.55 ± 20.89	0.034∗
PLT(10^9^/L)	245.63 ± 73.59	216.48 ± 58.40	0.038∗
PT (s)	10.62 ± 2.83	10.72 ± 2.10	0.032∗
PTA (%)	117.20 ± 20.92	108.96 ± 18.64	0.042∗
Na^+^ (mmol/L)	140.01 ± 3.65	141.30 ± 1.70	0.020∗
TG (mmol/L)	1.56 ± 0.94	1.34 ± 0.97	0.026∗
LDL (mmol/L)	2.66 ± 0.89	2.32 ± 0.77	0.048∗
BNP (pg/ml)	187.67 ± 164.89	149.24 ± 154.06	0.047∗
LVEDD (mm)	41.47 ± 9.70	45.48 ± 7.79	0.045∗
EF (%)	65.31 ± 8.16	68.10 ± 6.66	0.037∗

Note: Compared with the two groups, ∗*P* < 0.05. The same below.

**Table 2:** Binary logistic regression analysis of blood stasis and physical and chemical indexes.

Independent variable	Coefficient value	Standard error	Wald *X*^2^	*P*	OR	95% confidence interval	
						Upper limit	Lower limit
HGB	− 0.040	0.019	4.581	0.032∗	0.961	0.926	0.997
PT	0.433	0.201	4.625	0.032∗	1.542	1.039	2.288
PTA	0.056	0.024	5.621	0.018∗	1.058	1.010	1.108
EF	− 0.181	0.081	4.131	0.042∗	0.835	0.701	0.994

**Table 3:** Factors of physical and chemical indexes related to qi depression.

	Qi depression (*n* = 137)	Non-qi depression (*n* = 63)	*P*
APTT(s)	26.89 ± 7.53	29.25 ± 9.16	0.022∗
TG (mmol/L)	1.49 ± 1.04	1.60 ± 0.70	0.048∗
TC (mmol/L)	4.55 ± 1.27	4.92 ± 1.13	0.048∗
LDL (mmol/L)	2.52 ± 0.88	2.80 ± 0.85	0.041∗
LDL (mmol/L)	2.52 ± 0.88	2.80 ± 0.85	0.041∗
LVESD (mm)	27.75 ± 3.81	28.81 ± 3.67	0.026∗
FS (%)	38.82 ± 5.20	36.91 ± 4.59	0.005∗

**Table 4:** Regression analysis results of qi depression and physical and chemical indexes.

Independent variable	Coefficient value	Standard error	Wald *X*^2^	*P*	OR	95% confidence interval upper limit lower limit	
APTT	-0.45	0.021	4.620	0.032∗	0.956	0.917	0.996
TC	− 0.304	0.133	5.193	0.023∗	0.738	0.568	0.958
FS	0.097	0.034	8.392	0.004∗	1.102	1.032	1.177

**Table 5:** Factors of physical and chemical indexes related to Qi deficiency.

	Qi deficiency (*n* = 94)	Non-Qi deficiency (*n* = 106)	*P*
HGB (g/L)	106.66 ± 18.99	134.43 ± 15.64	0.000∗
APTT (s)	28.90 ± 7.59	26.51 ± 8.46	0.022∗
K^+^ (mmol/L)	4.01 ± 0.42	4.12 ± 0.37	0.048∗
BNP (pg/ml)	206.12 ± 180.64	160.08 ± 144.04	0.043∗
LVEDD (mm)	34.89 ± 8.08	48.48 ± 5.16	0.000∗∗
LAD (mm)	36.20 ± 4.55	34.32 ± 5.97	0.012∗

**Table 6:** Regression analysis results of qi deficiency and physical and chemical indexes.

Independent variable	Coefficient value	Standard error	Wald *X*^2^	*P*	OR	95% confidence interval upper limit lower limit	
HGB	− 0.095	0.020	23.660	0.000∗	0.909	0.875	0.945
LVEDD	− 0.389	0.078	24.965	0.000∗	0.678	0.582	0.790
LAD	0.147	0.054	7.302	0.007∗	1.159	1.041	1.289

**Table 7:** Factors of physical and chemical indexes related to yin deficiency.

	Yin deficiency (*n* = 85)	Non-Yin deficiency (*n* = 115)	*P*
HGB (g/L)	113.14 ± 21.38	127.47 ± 20.78	0.000∗
APTT (s)	29.47 ± 7.76	26.28 ± 8.16	0.001∗
CKMB (u/L)	12.19 ± 6.37	16.10 ± 14.76	0.048∗
LVEDD (mm)	37.62 ± 9.98	45.40 ± 7.68	0.000∗
LVPW (mm)	9.79 ± 1.07	9.37 ± 0.96	0.021∗

**Table 8:** Regression analysis results of yin deficiency and physical and chemical indexes.

Independent variable	Coefficient value	Standard error	Wald *X*^2^	*P*	OR	95% confidence interval upper limit lower limit	
APTT	0.060	0.022	7.277	0.007∗	1.062	1.017	1.109
CKMB	− 0.065	0.026	6.323	0.012∗	0.937	0.890	0.986
LVEDD	− 0.089	0.023	15.596	0.000∗	0.915	0.875	0.956
LVPW	0.673	0.186	13.096	0.000∗	1.961	1.362	2.824

**Table 9:** Factors of physical and chemical indexes related to phlegm turbidity.

	Phlegm turbidity (*n* = 54)	Non-phlegm turbidity (*n* = 146)	*P*
HGB (g/L)	127.50 ± 20.46	119.12 ± 22.39	0.018∗
PLT (10^9^/L)	223.72 ± 68.89	247.54 ± 72.42	0.038∗
APTT (s)	24.55 ± 9.74	28.78 ± 7.15	0.021∗
ALT (u/L)	19.68 ± 11.61	23.83 ± 13.56	0.023∗
AST (u/L)	18.83 ± 7.77	21.98 ± 8.33	0.034∗
Cl^−^ (mmol/L)	105.21 ± 3.31	103.98 ± 8.86	0.030∗
LVEDD (mm)	45.65 ± 7.98	40.78 ± 9.74	0.001∗
FS (%)	36.02 ± 6.43	39.03 ± 4.23	0.002∗

**Table 10:** Regression analysis results of phlegm turbidity and physical and chemical indexes.

Independent variable	Coefficient value	Standard error	Wald *X*^2^	*P*	OR	95% confidence interval upper limit lower limit	
ALT	− 0.034	0.017	4.186	0.041∗	0.966	0.935	0.999
APTT	− 0.056	0.025	4.997	0.025∗	0.946	0.901	0.993
LVEDD	0.062	0.021	9.029	0.003∗	1.064	1.022	1.108
FS	− 0.105	0.037	8.323	0.004∗	0.900	0.838	0.967

**Table 11:** Factors of physical and chemical indexes related to qi stagnation.

	Qi stagnation (*n* = 52)	Non-Qi stagnation (*n* = 148)	*P*
WBC (10^9^/L)	6.38 ± 1.66	5.78 ± 1.65	0.005∗
HGB (g/L)	131.73 ± 19.73	117.74 ± 21.86	0.000∗
PT (s)	12.23 ± 4.67	10.08 ± 1.11	0.041∗
FIB (g/L)	2.54 ± 0.62	2.89 ± 1.06	0.049∗
HDL (mmol/L)	1.30 ± 0.34	1.75 ± 3.33	0.010∗
BNP (pg/ml)	129.16 ± 122.40	200.19 ± 172.23	0.006∗
LVEDD (mm)	46.42 ± 7.25	40.57 ± 9.78	0.000∗
LAD (mm)	33.48 ± 6.63	35.81 ± 4.80	0.023∗

**Table 12:** Regression analysis results of qi stagnation and physical and chemical indexes.

Independent variable	Coefficient value	Standard error	Wald *X*^2^	*P*	OR	95% confidence interval upper limit lower limit	
WBC	0.288	0.119	5.877	0.015∗	1.333	1.057	1.682
PT	0.335	0.093	12.923	0.000∗	1.398	1.165	1.678
BNP	− 0.004	0.002	6.728	0.009∗	0.996	0.993	0.999
FIB	− 0.705	0.258	7.467	0.006∗	0.494	0.298	0.819
LVEDD	0.074	0.023	10.206	0.001∗	1.077	1.029	1.126
LAD	− 0.102	0.037	7.526	0.006∗	0.903	0.840	0.971

## Data Availability

The data used to support this study are available from the corresponding author upon request.
